# Mathematical Modeling and Computational Prediction of High-Risk Types of Human Papillomaviruses

**DOI:** 10.1155/2022/1515810

**Published:** 2022-07-21

**Authors:** Junchao Zhang, Kechao Wang

**Affiliations:** Department of Mathematics, Harbin University, Harbin, Heilongjiang 150001, China

## Abstract

Cervical cancer is one of the main causes of cancer death all over the world. Most diseases such as cervical epithelial atypical hyperplasia and invasive cervical cancer are closely related to the continuous infection of high-risk types of human papillomavirus. Therefore, the high-risk types of human papillomavirus are the key to the prevention and treatment of cervical cancer. With the accumulation of high-throughput and clinical data, the use of systematic and quantitative methods for mathematical modeling and computational prediction has become more and more important. This paper summarizes the mathematical models and prediction methods of the risk types of human papillomavirus, especially around the key steps such as feature extraction, feature selection, and prediction algorithms. We summarized and discussed the advantages and disadvantages of existing algorithms, which provides a theoretical basis for follow-up research.

## 1. Introduction

Human papillomavirus (HPV) usually causes benign papillomas and epithelial malignancies [1]. About 30 years ago, researchers found a close relationship between HPV and cervical cancer. Since then, specific HPV type DNA has been found in almost all cervical cancer biopsies [2]. Epidemiological studies also continue to show that HPV is the main cause of cervical cancer. HPV is a papillomavacuolar virus of the family lactomaviridae. It is a spherical DNA virus with 72 shell particles on the surface, a 20 hedral three-dimensional symmetrical nucleocapsid structure, with a diameter of about 45-55 nm [3]. It contains 8000 base pairs, of which 88% are viral proteins. According to the function of HPV genome, it can be divided into three parts: noncoding region, early gene region, and late gene region. The noncoding regions include promoters, enhancers, and silencers, which play an important role in DNA replication and transcriptional regulation. The early gene region contains six genes E1, E2, E4, E5, E6, and E7, including proteins and oncogenes required in the process of replication [4]. The late gene region contains L1 and L2 genes, which encode the structural proteins that constitute the virus capsid [5].

The early region encodes and produces six proteins. Their functions are as follows: E1 protein mainly controls virus replication and replication inhibition and is expressed in the early stage of virus infection; E2 protein is a specific DNA binding protein [6], which can not only regulate mRNA transcription and DNA replication but also inhibit the expression of E6 and E7 proteins; E4 protein is expressed during virus infection and plays an important role in virus replication and mutation; E5 protein is the smallest transforming protein [7]. It consists of two functional regions, one is the amino terminal hydrophobic region, which is related to the insertion position of E5 protein on the membrane, and the other is the hydrophilic region of carboxyl terminal. If the carboxyl terminal is injected into resting cells, it can induce cell DNA synthesis. In addition, it can also induce the expression of a variety of oncogenes; E6 and E7 proteins are the two most important proteins. They can not only regulate the cell cycle [8] but also play an important role in the proliferation of cancer cells.

More than 200 HPV types have been identified, and about 40 types can invade the female reproductive tract [9]. When the identified HPV has significant homology differences with the defined HPV types, some new types will be defined. Epidemiological studies have shown that there is a strong relationship between reproductive human papillomavirus and cervical cancer, which is not related to other risk factors. According to its relative malignancy, HPV can be divided into two or three types: low-risk type, medium-risk type, and high-risk type. The high-risk HPVs include HPV16, 18, 31, 33, 34, 35, 39, and 45, and the low-risk HPVs include HPV6, 11, 42, 43, and 44 [10–13].

The distribution of HPV types has obvious geographical characteristics. Research shows that among the high-risk types worldwide, HPV16 accounts for 51% [14], followed by HPV16, accounting for 16%, others, such as HPV45 accounts for 9%, HPV31 accounts for 6%, and HPV33 accounts for 3%. The sum of these four common HPV types exceeds 80%. However, in Latin America, HPV33 is the most common, followed by HPV39 and 59. In Asia, in addition to the most common HPV16 and 18 [15], HPV 52 and 58 account for far more cervical cancer than Western and African countries.

Different types of HPV have different clinical manifestations. According to the tissues invaded, HPV can be divided into high (low) risk type of skin and high (low) risk type of mucosa [16]. Low-risk skin types such as HPV1, 2, 3, and 4 are generally related to common warts, flat warts, and other diseases. High-risk skin types such as HPV5, 8, 14, and 17 are associated with anal cancer, prostate cancer, bladder cancer, and so on. For low-risk types of mucosa: HPV6, 11, 13, 32, 34, 40, 42, etc., they are generally related to diseases such as genital, anal, oropharyngeal, and esophageal mucosal infection. Mucosal high-risk types such as HPV16, 18, 30, 31, 33, 35, and 39 can lead to cervical cancer, rectal cancer, tonsillar cancer, and other diseases [17].

Now, there are many epidemiological and experimental methods to identify HPV types [18–21]. They mainly use polymerase chain reaction (PCR) technology to realize the rapid detection of clinical samples. With the rapid accumulation of human papillomavirus data, a reliable and effective calculation method is needed to predict high-risk HPV. In recent years, many computational models have been proposed to predict HPV high-risk types. Eom et al. designed genetic algorithm to predict HPV type through the sequence fragment distribution characteristics of HPV [22]. Joung et al. designed the prediction method of HPV type based on support vector machine prediction and hidden Markov model [23, 24]. Through systematic analysis, Park et al. suggested using decision tree to construct the typing model of human papillomavirus [25]. Kim and Zhang calculated the distance distribution of amino acid pairs and further predicted the risk type of HPV through E6 protein [26, 27]. Kim et al. extracted the differential features of protein secondary structure and designed a set of support vector machine (GSVM) to classify HPV types [28]. Esmaeili et al. calculated Chou's pseudoamino acid composition of HPV sequence and classified HPV types using ROC [29]. Alemi et al. systematically compared the physical and chemical properties of high-risk and low-risk HPV and build a prediction model of high-risk HPV based on the support vector machine [30]. Wang et al. used protein “sequence space” to explore this information to predict high-risk types of HPVs [31]. Xu et al. proposed a HPV high-risk prediction model based on reduced amino acids, and they divided 20 amino acids into several nonoverlapping groups and calculated the structure and chemical patterns of each group as the basis for distinguishing high-risk HPV [32].

In this paper, we introduce the development of HPV typing in cervical cancer, mainly focusing on sequence characteristics and predicted secondary structure characteristics. The feature fusion method and feature selection algorithm are discussed. Finally, we review the multiple classification and various machine learning algorithms in HPV typing of cervical cancer.

## 2. Benchmark Datasets

HPV database is from Los Alamos National Laboratory (LANL), with a total of 72 HPV types. HPV risk types were manually determined based on the HPV profile [33]. If HPV belongs to skin related or skin group, HPV is classified as a low-risk type. On the other hand, it is classified as a high-risk type if HPV is known to be a high-risk type of cervical cancer [28]. Some researchers may build their own HPV dataset from SWISS-PROT. For these sequences, some researchers will complete their own wonderful processing. Here, we focus on using mathematical models to detect the risk types of human papillomavirus. Therefore, the detailed processing of data sets is no longer our important discussion content.

## 3. Methods

### 3.1. Feature Extraction

The extraction of HPV sequence information is transforming from complex structure to extraction of mathematical features [34]. Directly extracting information from the complex structure of HPV protein will cause large errors, and the extracted information may not be comprehensive. However, it is very easy to directly extract the mathematical features from the protein sequence, there is no influence of error on the connection, and the extracted information contains all the protein information.

#### 3.1.1. Sequence Features

*(1) K-Mer*. Protein sequences and peptides can be regarded as a set of signs [35], and we can analyze their characteristics through the frequency of k-mer to obtain the difference between the two HPV sequences. If *k* is 1, it means that it is the composition of amino acids, which is calculated as follows [36]:

(1) $$\begin{array}{c} F\left(S\right)={\left(f_{1},f_{2},\cdots ,f_{20}\right)}^{T}, \end{array}$$

(2) $$\begin{array}{c} f_{i}=\frac{n_{i}}{\sum_{i=1}^{20}n_{i}}, \end{array}$$

where *n*_*i*_ means the number of the amino acid *i* in the protein sequence.

*(2) Order-Based Features*. Order-based features reflect the physical and chemical interaction among the amino acids pairs, which can be described by sequence coupling score and quasisequence score [37].

Suppose *S* is a protein sequence with a length of *L*, *τ*_*j*_ is denoted as the sequence interaction factor describing the sequence influence:

(3) $$\begin{array}{c} \tau_{j}=\frac{1}{L-j}\overset{L-j}{\underset{i=1}{\sum }}J_{i,i+j}\left(j=1,2,\cdots ,k,k<L\right), \end{array}$$

where *J*_*i*,*i*+*j*_ is the physical and chemical distance between the amino acid *Ri* and *R*_*i*+*j*_, which can be calculated:

(4) $$\begin{array}{c} J_{i,i+j}=D^{2}\left(R_{i},R_{i+\text{j}}\right). \end{array}$$

The calculation method of *D*^2^ can consider the hydrophobicity value, polarity value, and side chain volume of amino acids. Thus, *S* can be defined by the following features:

(5) $$\begin{array}{c} V_{QSOE}\left(S\right)={\left[v_{1},v_{2},\cdots ,v_{20},v_{20+1},\cdots ,v_{20+k}\right]}^{T}. \end{array}$$

The first 20 features are k-mer features, and the latter *k*-dimensional features represent the interaction information of amino acid sequences.

*(3) Amino Acid Distribution*. Amino acid distribution is composed of amino acid composition, transformation, and distribution. This component can be regarded as the amino acid component of HPV, which can be original sequence or reduced sequence to describe the sequence component [38]. The transformation can be described by calculating the number of conversions between a base and a subsequent base. It can be calculated by the following formula:

(6) $$\begin{array}{c} Trs=\frac{{\text{Count}}_{rs}+{\text{Count}}_{sr}}{N-1}, \end{array}$$

where *N* is the number of amino acids, and Count_*sr*_ is the number of conversions between the base *s* and a subsequent base *r*.

*(4) Pseudoamino Acid Composition (PseAAC)*. In order to avoid the loss of many important information hidden in HPV sequences, Chou proposed pseudoamino acid composition (PseAAC), which is not a simple AAC to represent protein samples [39]. Pseudoamino acid composition is a vector with size *R* + *λ*, where *R* is the composition size of the amino acids, and the latter *λ* dimension is the information of pseudoamino acid composition [29]. They can be calculated by the following formula:

(7) $$\begin{array}{c} v_{u}=\left\{\begin{array}{c} \frac{f_{u}}{\sum_{u=1}^{R}f_{u}+w\sum_{k=1}^{\lambda }\tau_{k}}\left(u\leq R\right),\\ \frac{w\tau_{u-20}}{\sum_{u=1}^{R}f_{u}+w\sum_{k=1}^{\lambda }\tau_{k}}\left(R\leq u\leq R+\lambda \right), \end{array}\right. \end{array}$$

where *f*_*u*_ is the frequency of RedAA, *w* is the weight, and *τ*_*k*_ can be calculated by the following formula:

(8) $$\begin{array}{c} \tau_{k}=\frac{1}{L-k}\overset{L-k}{\underset{i=1}{\sum }}J_{i,j+k}\left(k<L\right), \end{array}$$

(9) $$\begin{array}{c} J_{i,j+k}=\frac{1}{3}\left\{{\left[H_{1}\left(R_{i}\right)-H_{1}\left(R_{i+k}\right)\right]}^{2}+{\left[H_{2}\left(R_{i}\right)-H_{2}\left(R_{i+k}\right)\right]}^{2}+{\left[M\left(R_{i}\right)-M\left(R_{i+k}\right)\right]}^{2}\right\}. \end{array}$$

*H*_*i*_(*R*_*i*_) represents molecular weight of amino acid residue *R*_*i*_, and *M*(*R*_*i*_) is the molecular weight of amino acid residue *R*_*i*_. Then, the protein sequence can be mapped to the following feature vectors by this way:

(10) $$\begin{array}{c} V_{\text{PseAAC}}\left(S\right)={\left[v_{1},v_{2},\cdots ,v_{20},\cdots ,v_{20+\lambda }\right]}^{T}. \end{array}$$

#### 3.1.2. Evolutionary Profile

*(1) Position Specific Scoring Matrix (PSSM)*. PSSM is developed on the basis of position frequency matrix [40], which can quantitatively describe the evolutionary characteristics of HPV sequences. At present, it is the most commonly used matrix feature model, especially for protein structural class prediction [41]. When a protein s with length *L* is given, its PSSM is defined as

(11) $$\begin{array}{c} \text{PSS}{\text{M}}_{s}=\left[\begin{array}{cccccc} P_{1⟶1} & P_{1⟶2} & \cdots & P_{1⟶j} & \cdots & P_{1⟶20}\\ P_{2⟶1} & P_{2⟶2} & \cdots & P_{2⟶j} & \cdots & P_{2⟶20}\\ \vdots & \vdots & \vdots & \vdots & \vdots & \vdots \\ P_{i⟶1} & P_{i⟶2} & \cdots & P_{i⟶j} & \cdots & P_{i⟶20}\\ \vdots & \vdots & \vdots & \vdots & \vdots & \vdots \\ P_{L⟶1} & P_{L⟶2} & \cdots & P_{L⟶j} & \cdots & P_{L⟶20} \end{array}\right], \end{array}$$

where *i*⟶*j* represents that the residue at the position of *i* − th mutated into the type of *j* during the course of biological evolution. *P*_*i*⟶*j*_ indicates the score of mutation, and the ordered 20 amino acids are marked as 1, 2, 3… 20. The close evolutionary relationship among these HPV sequences can be described by their PSSM [42]. We search homogeneous sequences from SWISS-PROT database with help of PSI-BLAST [43–45] and normalize PSSM using the following sigmoid function:

(12) $$\begin{array}{c} f\left(x\right)=\frac{1}{1+e^{-x}}. \end{array}$$

*(2) Structural Properties of PSSM*. When [0, *L* − 1] × ∑⟶*ℜ* is used to describe a function *M*, *L* is the length of a function *M*. The PSSM of the sequence *Seq*_0_ will be transformed into a RedPSSM of its reduced sequence *Seq*_*s*_,

(13) $$\begin{array}{c} \left[0,L\right]\times \underset{Seq_{0}}{\sum }⟶\left[0,L\right]\times {\underset{Seq}{\sum }}_{r}, \end{array}$$

where ∑_*Seq*_0__ and ∑_*Seq*_*r*__ are finite alphabet sets of the original and reduced sequences. [RedPSSM]_*ij*_ is defined as

(14) $$\begin{array}{c} {\left[\text{RedPSSM}\right]}_{ij}=\overset{g_{s}\left(j\right)}{\underset{j=1}{\sum }}\frac{P_{i⟶j}}{g_{s}\left(j\right)}, \end{array}$$

where *g*_*s*_(*j*) represents the size of the reduced group which is made up with the reduced amino acid *j*, and *j* belongs to 1 ≤ *j* ≤ |∑_*seq*_*r*__|.

Auto covariance (AC) is a correlation factor, which has been widely used in various fields of bioinformatics [46]. It can connect adjacent residues according to protein sequence and convert PSSM into equal length vector [47]. The AC variable can represent the average interaction between residues with a series of lags, which is defined as

(15) $$\begin{array}{c} AC_{j,g}\left(S\right)=\frac{1}{L-g}\overset{L-g}{\underset{i=1}{\sum }}\left(P_{i,j}-{\bar{P}}_{j}\right)\left(P_{i,j+g}-{\bar{\text{P}}}_{j}\right), \end{array}$$

where *AC*_*j*,*g*_(*S*) can indicate the interaction between two spacer *g* residues. But it can just calculate the residue interaction in the same column [48]. In order to solve this problem, we calculated total correlations among all the columns by the following formula:

(16) $$\begin{array}{c} \text{RA}{\text{C}}_{g}\left(h,j\right)=\frac{1}{L-g}\overset{L-g}{\underset{i=1}{\sum }}\left|{\left[\text{RedPSSM}\right]}_{i,h}-\frac{{\left[\text{RedPSSM}\right]}_{i,h}+{\left[\text{RedPSSM}\right]}_{i+g,j}}{2}\right|\times \left|{\left[\text{RedPSSM}\right]}_{i+g,h}-\frac{{\left[\text{RedPSSM}\right]}_{i,h}+{\left[\text{RedPSSM}\right]}_{i+g,j}}{2}\right|=\frac{1}{4\left(L-g\right)}\overset{L-g}{\underset{i=1}{\sum }}{\left({\left[\text{RedPSSM}\right]}_{i,h}-{\left[\text{RedPSSM}\right]}_{i+g,h}\right)}^{2}. \end{array}$$

#### 3.1.3. Secondary Structure Features

In order to improve the accuracy of HPV high-risk types, some researchers analyzed the protein secondary structures of HPV, extracted its characteristics, and constructed prediction models [28, 49]. Given a protein sequence, we predict its secondary structure sequence. Its secondary structure content (content_SE_) can be calculated as

(17) $$\begin{array}{c} \text{conten}{\text{t}}_{\text{SE}}=\frac{\text{Coun}{\text{t}}_{\text{SE}}}{\sum_{x\in \left\{C,H,E\right\}}\text{C}\text{oun}{\text{t}}_{x}}, \end{array}$$

where  SE belong to  {*C*, *H*, *E*}. *H* is *α*-helix, *E* is *β*-strand, and *C* is coil. Gk and Herand calculated the first and second order composition moment vector (CMV) as the structure features [50], which is defined as the following formula:

(18) $$\begin{array}{c} \text{CM}{\text{V}}_{\text{SE}}^{k}=\frac{\sum_{j=1}^{\text{Coun}{\text{t}}_{\text{SE}}}\text{P}{\text{O}}_{\text{SE}j}^{k}}{\prod_{d=1}^{k}\left(N-d\right)}, \end{array}$$

wherePO_SE*j*_ represents the element at position *j* in the secondary structure sequence with length *N*, which *k* is the vector order.

In order to further study the arrangement of different structural elements, some important structural fragments or patterns have been proposed one after another [51]. The length of the longest segment (MaxSeg_SE_) is defined as the following formula:

(19) $$\begin{array}{c} \text{MaxSe}{\text{g}}_{\text{SE}}=\text{MaxLen}\left(\text{SEG}:\text{SE}{\text{G}}_{\text{SE}}\right), \end{array}$$

where MaxLen represents the function of the maximal segment length, and SEG_SE_ is the composed of each segment of the structure element SE [52]. In order to reduce the length effect, a normalized length of the longest segment (NMaxSeg_SE_) is defined

(20) $$\begin{array}{c} N\text{MaxSe}{\text{g}}_{\text{SE}}=\frac{\text{MaxLen}\left(\text{SEG}:\text{SE}{\text{G}}_{\text{SE}}\right)}{N}, \end{array}$$

where *N* is the sequence length. In addition to the maximal segment length, the average length of the segment (AvgSeg_SE_) is also an important feature of protein secondary structure, which is defined as

(21) $$\begin{array}{c} \text{AvgSe}{\text{g}}_{\text{SE}}=\frac{\sum \text{L}\text{en}\left(\text{SEG}:\text{SE}{\text{G}}_{\text{SE}}\right)}{\text{Conten}{\text{t}}_{\text{SE}{\text{G}}_{\text{SE}}}}, \end{array}$$

where Content_SEG_SE__ represents the substance of SEG_SE_, and Len is a function of segment length. The normalized average length of the segment (NAvgSeg_SE_) is

(22) $$\begin{array}{c} N\text{AvgSe}{\text{g}}_{\text{SE}}=\frac{\sum \text{L}\text{en}\left(\text{SEG}:\text{SE}{\text{G}}_{\text{SE}}\right)}{\text{Conten}{\text{t}}_{\text{SE}{\text{G}}_{\text{SE}}}\times N}, \end{array}$$

where *N* represents the length of protein sequence.

Zhang et al. analyzed the secondary structure of protein, only considered the helical and folded structural units, ignoring the irregular curl [53]. According to this simplification rule, they got a simplified protein secondary structure sequence and defined the transition probability matrix (TPM) as follows:

(23) $$\begin{array}{c} \text{TPM}=\left(\begin{array}{cc} p_{\alpha \alpha } & p_{\alpha \beta }\\ p_{\beta \alpha } & p_{\beta \beta } \end{array}\right), \end{array}$$

where

(24) $$\begin{array}{c} p_{a_{i}a_{j}}=\left\{\begin{array}{cc} \frac{\text{Conten}{\text{t}}_{a_{i}a_{j}}}{\sum_{t=1}^{2}\text{C}\text{onten}{\text{t}}_{a_{i}a_{t}}}\; & \overset{2}{\underset{t=1}{\sum }}\text{C}\text{onten}{\text{t}}_{a_{i}a_{t}}\neq 0,\\ 0 & \overset{2}{\underset{t=1}{\sum }}\text{C}\text{onten}{\text{t}}_{a_{i}a_{t}}=0, \end{array}\right. \end{array}$$

where *a*_*i*_ belongs to {*α*, *β*}, *a*_*i*_ is followed by the *a*_*j*_, and the size of the event is described by Content_*a*_*i*_*a*_*j*__.

Most researchers pay attention to the content of structural units, so sometimes they do not know the location information of these structural units in the protein structure. Dai et al. proposed some location-based structural features [54]. If the distance Dis(*δ*) of the given structural element *δ* is 1, they will be divided into a structural domain. If not, they will be divided into two different structural domains. If the Dis(*δ*) is given, its probability distribution can be achieved. The definitions of digital feature semimean Semi − *E*_(*k*)_(*δ*) and semivariance Semi − *D*_(*k*)_(*δ*) are as follows:

(25) $$\begin{array}{c} \text{Semi}-E_{\left(k\right)}\left(\delta \right)=\overset{k}{\underset{Dis\left(\delta \right)=1}{\sum }}\text{D}\text{is}\left(\delta \right)\times P\left(\text{Dis}\left(\delta \right)\right), \end{array}$$

(26) $$\begin{array}{c} \text{Semi}-D_{\left(k\right)}\left(\delta \right)=\overset{k}{\underset{\text{Dis}\left(\delta \right)=1}{\sum }}{\left(\text{Dis}\left(\delta \right)\right)}^{2}\times P\left(\text{Dis}\left(\delta \right)\right)-{\left[\overset{k}{\underset{\text{Dis}\left(\delta \right)=1}{\sum }}\text{D}\text{is}\left(\delta \right)\times P\left(\text{Dis}\left(\delta \right)\right)\right]}^{2}. \end{array}$$

The ratio of the standard Semi − *D*_(5)_ to Semi − *E*_(5)_ can be calculated by:

(27) $$\begin{array}{c} \text{PSSF}\left(\delta \right)=\frac{\text{Semi}-E_{\left(5\right)}\left(\delta \right)}{\sqrt{\text{Semi}-D_{\left(5\right)}\left(\delta \right)}}. \end{array}$$

PSSF(*δ*) is used to describe the position distribution of predicted secondary structural elements.

### 3.2. Feature Selection

Feature selection (SF) is one of the important steps in data processing, which plays an important role in data mining, pattern recognition, and machine learning [32]. It solves the problem of how to select the input features corresponding to the optimal prediction results. Through feature selection, the complexity of the problem can be reduced, and the prediction accuracy, robustness, and interpretability of the learning algorithm can be improved [55]. Therefore, feature selection can be used to select the characteristics of HPV risk types [56]. More importantly, it helps to have a deeper understanding of HPV sequences when we analyze their characteristics. This section summarizes some feature selection methods.

#### 3.2.1. Mutual Information

The feature selection method based on mutual information can capture the nonlinear relationship between variables, which is more suitable for dealing with complex classification problems [57]. Mutual information can be expressed as characteristic matrix *X*, and the relevant category is *C*. Mutual information can be defined as

(28) RelXi=IXi;C=∑Xi,CPXi,ClogPXi,CPXiPC.

When the set of *S* is selected, the redundant formula Eq. (29) is

(29) $$\begin{array}{c} \text{Red}\left(\left.X_{i}\right|S\right)=\frac{1}{S}\underset{X_{j}\in S}{\sum }I\left(X_{i};X_{j}\right). \end{array}$$

As can be seen from the above definition, mutual information aims to select the features that are most relevant to the target category and have the least redundancy between the selected features [58]. Therefore, feature selection can be realized directly according to the value of mutual information.

#### 3.2.2. Support Vector Machine Recursive Feature Elimination (SVM-RFE)

Support vector machine has been widely used in the field of pattern recognition and is very suitable for small samples with high-dimensional data. SVM-RFE is a sequential reverse selection (SBS) algorithm based on the maximum interval principle of SVM [59]. SVM-RFE can be divided into linear SVM-RFE and nonlinear SVM-RFE.

*(1) Linear SVM-RFE*. There is a training sample set {*xi*, *yi*}, *yi* ∈ {−1, 1}, *i* = 1, 2, ⋯, *n*. The linear SVM can be calculated by the following formula:

(30) $$\begin{array}{c} f\left(x\right)=a\cdot x+b, \end{array}$$

where *a* is the weight vector of the optimal hyperplane, and *b* is the threshold.

By introducing Lagrange's formula, the optimization problem of SVM can be transformed into the following dual programming problem:

(31) $$\begin{array}{c} L_{D}=\overset{n}{\underset{i=1}{\sum }}\alpha_{i}-\frac{1}{2}\overset{n}{\underset{i,j=1}{\sum }}\alpha_{i}\alpha_{j}y_{i}y_{j}x_{i}x_{j}, \end{array}$$

where *α*_*i*_ can be calculated by solving the maximum value of *L*_*D*_ under the range of *α*_*i*_ ≥ 0 and ∑_*i*=1_^*n*^*α*_*i*_*y*_*i*_ = 0. So *a* Eq. (32) can be defined as follows:

(32) $$\begin{array}{c} a=\overset{n}{\underset{i=1}{\sum }}\alpha_{i}y_{i}x_{i}. \end{array}$$

The ranking criterion score of the *k*-th feature is defined as the following equation:

(33) $$\begin{array}{c} J\left(k\right)=w_{k}^{2}. \end{array}$$

During the training process, the feature with the smallest score of the ranking criterion is removed, and the remaining features are used to train the SVM for the next iteration.

*(2) Nonlinear SVM-RFE*. When the sample size is larger than the number of features, nonlinear SVM-RFE can obtain better results [60]. Features can be mapped to new spaces in higher dimensions by nonlinear SVM-RFE:

(34) $$\begin{array}{c} x\in R^{d}\mapsto \varphi \left(x\right)\in R^{h}. \end{array}$$

After being mapped to the new space, the samples can be divided into linear features. It can be calculated by the formula of Lagrangian:

(35) $$\begin{array}{c} L_{D}=\overset{n}{\underset{i=1}{\sum }}\alpha_{i}-\frac{1}{2}\overset{n}{\underset{i,j=1}{\sum }}\alpha_{i}\alpha_{j}y_{i}y_{j}\varphi \left(x_{i}\right)\varphi \left(x_{j}\right). \end{array}$$

Here, *Φ*(*x*_*i*_)*Φ*(*x*_*j*_) can be changed into a Gaussian kernel formula *K*(*x*_*i*_, *x*_*j*_):

(36) $$\begin{array}{c} K\left(xi,xj\right)=\ell^{-\lambda {\left|\left|x_{i}-x_{j}\right|\right|}^{2}}. \end{array}$$

The ranking criteria of feature *k* can be described by the following formula:

(37) $$\begin{array}{c} J\left(k\right)=\frac{1}{2}\overset{n}{\underset{i,j=1}{\sum }}\alpha_{i}\alpha_{j}y_{i}y_{j}K\left(x_{i},x_{j}\right)-\frac{1}{2}\overset{n}{\underset{i,j=1}{\sum }}\alpha_{i}\alpha_{j}y_{i}y_{j}K\left(x_{i}^{\left(-k\right)},x_{j}^{\left(-k\right)}\right), \end{array}$$

where *x*_*i*_^(−*k*)^ represents that k has been dropped.

#### 3.2.3. Genetic Algorithm

Genetic algorithm is an adaptive search strategy, and its principle is similar to the survival mechanism of the fittest in nature [61]. It has strong adaptability, strong independence of domain knowledge, and can carry out a large number of parallel computing. Therefore, it is more suitable for processing large-scale complex data, especially for solving multiobjective optimization problems [62]. Given an HPV data set, we construct its characteristic matrix *X* and use genetic algorithm to obtain an eigenvector, which is an optimal feature set [63].

#### 3.2.4. Kurtosis and Skewness

Kurtosis and skewness are two characteristics describing distribution [64], which can distinguish the distribution of different characteristics. Therefore, many studies calculated the skewness and kurtosis of each feature and selected certain features according to the value of skewness and kurtosis. Given the distribution of a feature {*x*_1_, *x*_2_, ⋯, *x*_*n*_}, its kurtosis and skewness are defined as follows:

(38) $$\begin{array}{c} \text{Kurtosis}=\frac{\sum_{i=1}^{n}{\left(x_{i}-\bar{x}\right)}^{4}}{\left(n-1\right)SD^{4}}-3, \end{array}$$

(39) $$\begin{array}{c} \text{Skewness}=\frac{\sum_{i=1}^{n}{\left(x_{i}-\bar{x}\right)}^{3}}{\left(n-1\right)SD^{3}}. \end{array}$$

#### 3.2.5. ReliefF Algorithm

ReliefF is an independent evaluation method, which evaluates each feature separately and assigns weight to the feature [65, 66]. For each time, it randomly selects a sample *R* from the training set and then calculates the latest instance from the same class *R* and different sample sets, and then the weight update rules in each step are as follows:

(40) $$\begin{array}{c} W\left(A\right)=W\left(A\right)-\overset{k}{\underset{j=1}{\sum }}\frac{\text{diff}\left(A,R,H_{j}\right)}{mk}+\underset{C\notin \text{class}\left(R\right)}{\sum }\frac{p\left(C\right)/1-p\left(\text{Class}\left(R\right)\right)\sum_{j=1}^{k}\text{d}\text{iff}\left(A,R,M_{j}\left(C\right)\right)}{mk}, \end{array}$$

where diff(*A*, *R*_1_, *R*_2_) represents the difference between the sample *R*_1_ and the sample *R*_2_ on the feature *A*, and *M*_*j*_(*C*) indicates the nearest neighbor of the position of *j* − th in class *C* Eq. (41). diff(*A*, *R*_1_, *R*_2_) can be calculated by the following formula:

(41) $$\begin{array}{c} \text{diff}\left(A,R1,R2\right)=\left\{\begin{array}{c} \frac{\left|R_{1}\left[A\right]-R_{2}\left[A\right]\right|}{\max\left(A\right)-\min\left(A\right)},\\ 0R_{1}\left[A\right]=R_{2}\left[A\right],\\ 1R_{1}\left[A\right]\neq R_{2}\left[A\right]. \end{array}\right. \end{array}$$

### 3.3. Prediction Algorithms

#### 3.3.1. Support Vector Machines (SVM)

SVM is a discriminant classifier, which is defined by the classification hyperplane [27]. In other words, the labeled training samples are used to train the model, and then the test sample classification is realized by outputting the best hyperplane [67]. When the prediction problem is nonlinear, the objective function of SVM can be defined as

(42) $$\begin{array}{c} f\left(x\right)=\overset{N}{\underset{i=1}{\sum }}\alpha_{i}y_{i}K\left(x_{i},x\right)+b, \end{array}$$

where *K*(*x*_*i*_, *x*) is a kernel function, *x*_*i*_ is a support vector, and *α*_*i*_ belongs to [0, *C*]. The Gaussian radial basis kernel function with strong learning ability and small error is often selected as the kernel function, which is defined as

(43) $$\begin{array}{c} K\left(x_{i},x\right)=\exp\left(-\frac{{\left\|x_{i}-x\right\|}^{2}}{2\sigma^{2}}\right), \end{array}$$

where *σ* is the coefficient of the kernel function and has high flexibility.

#### 3.3.2. Principal Component Analysis (PCA)

PCA is a statistical analysis method that converts multiple indicators into a few comprehensive indicators. The idea of PCA is to replace the original more with fewer comprehensive variables [68]. The first step of PCA is to normalize the matrix which can also be expressed as the following mathematical formula:

(44) $$\begin{array}{c} Zij=\frac{x_{ij}-{\bar{x}}_{j}}{s_{j}}\left(i=1,2,\cdots ,n;j=1,2,\cdots ,p\right), \end{array}$$

(45) $$\begin{array}{c} {\bar{x}}_{j}=\frac{\sum_{i=1}^{n}x_{ij}}{n},s_{j}^{2}=\frac{\sum_{i=1}^{n}{\left(x_{ij}-x_{j}\right)}^{2}}{n-1}. \end{array}$$

The second step of PCA is to obtain the correlation of coefficient matrix for *Z*:

(46) $$\begin{array}{c} R={\left[r_{ij}\right]}_{p}xp=\frac{Z^{T}Z}{n-1}, \end{array}$$

(47) $$\begin{array}{c} rij=\frac{\sum zkj\cdot zkj}{n-1}\left(i,j=1,2,\cdots ,p\right). \end{array}$$

#### 3.3.3. *K*-Nearest Neighbor Algorithm (KNN)

KNN is an important nonparametric classification method, which classifies the samples according to the categories of most *k*-nearest neighbor samples in the feature space [69]. However, the basic *k*-nearest neighbor classification algorithm needs global search, which has high computational complexity and slow computing speed. In order to reduce the influence of the same feature function in the traditional KNN algorithm, different weights can be assigned to the features in the distance formula to measure the similarity. For example, in Euclidean distance formula, different weights are assigned to different features, as shown in the formula:

(48) $$\begin{array}{c} d\left(X,Y\right)=\sqrt{\overset{n}{\underset{i=1}{\sum }}{\left(x_{i}-y_{i}\right)}^{2}}. \end{array}$$

#### 3.3.4. Partial Least Square Discriminant Analysis (PLS-DA)

PLS-DA is a standard high-dimensional data analysis method, and it is especially suitable for situations where there are a large number of explanatory variables [70], multicollinearity samples, few observations, and large interference noises. PLS-DA first treats the sample category with dummy variables which can be calculated by the following formula:

(49) $$\begin{array}{c} \left\{\begin{array}{c} Yk=1,Y=k\\ Yk=0,Y\neq k \end{array}\right.,\left(k=1,2,\cdots ,q\right), \end{array}$$

where *Y* represents categorical variables, and *q* is a dummy variable. The relationship model between explanatory variables, response variables is established by least square regression, and then, the category of each sample is determined by comparing the predicted values of model response variables. If the predicted value of the dummy variable component is the largest, it is determined that the sample belongs to the category corresponding to the dummy variable.

#### 3.3.5. Classification and Regression Tree (CART)

CART is a nonparametric statistical process of data analysis. Its characteristic is to make full use of the binary tree structure in the calculation process, that is, the root node contains all samples, and the root node is divided into two children under certain partition rules [71]. The process of node is repeated on the subbook point and becomes a regression process until it can no longer be divided into leaf nodes [72]. When all nodes can be classified into class *C* (*k* = 1, 2, ⋯, *C*), the Gini impurity of node *A* can be expressed by the following formula:

(50) $$\begin{array}{c} \text{Gini}\left(A\right)=1-\overset{C}{\underset{k=1}{\sum }}p_{k}^{2}, \end{array}$$

where *p*^*k*^ is the proportion of the sample which belongs to class *k*. If class *A* can be divided into *B* and *C*. The probability of *B* in the sample *A* is *p* and *C* is *q*. And the size of impurities will be expressed by the following formula:

(51) $$\begin{array}{c} \text{Gini}\left(A\right)-p\cdot \text{Gini}\left(B\right)-q\cdot \text{Gini}\left(C\right). \end{array}$$

#### 3.3.6. Linear Discriminant Analysis (LDA)

LDA is a statistical analysis method used to determine the type of sample [73], which has been widely used in the prediction of protein structural classes. By finding the feature vector *w*, the *k* sets of *m* metadata are mapped into another lower-dimensional direction. Then classify with the sample in the new space.

(52) $$\begin{array}{c} w_{opt}=\arg\underset{w}{\max}\frac{\left|w^{T}S_{B}w\right|}{\left|w^{T}S_{w}w\right|}. \end{array}$$

*S*_*B*_ is an interclass deviation matrix:

(53) $$\begin{array}{c} S_{B}=\sum \left({\text{m}}_{x}-m_{y}\right){\left(m_{x}-m_{y}\right)}^{T}. \end{array}$$

*S*_*w*_ is an intraclass deviation matrix:

(54) $$\begin{array}{c} S_{w}=\overset{N_{x}}{\underset{i=1}{\sum }}\left(x_{i}-m_{x}\right){\left(x_{i}-m_{x}\right)}^{T}+\overset{N_{y}}{\underset{i=1}{\sum }}\left(y_{i}-m_{y}\right){\left(y_{i}-m_{y}\right)}^{T}, \end{array}$$

where {*x*_*i*_, *i* = 1, 2, ⋯, *N*_*x*_} represents class *p*, {*y*_*i*_, *i* = 1, 2, ⋯, *N*_*y*_} represents class *n*. Where *m*_*x*_ and *m*_*y*_, respectively, represent the average of class *p* and class *n*.

#### 3.3.7. Extreme Gradient Boosting (XGBoost)

The gradient boosting algorithm framework supports a variety of different loss functions [74]. In addition to the exponential loss function, it also includes the mean square error loss function and logarithmic loss function. XGBoost algorithm is an enhanced version of gradient boosting algorithm. It is more efficient, flexible, and portable [75]. It used the training data *x*_*i*_ to predict a target variable *y*_*i*_.

First of all, the objective function can be calculated as

(55) $$\begin{array}{c} obj=\Sigma_{1=1}^{n}l\left(y_{i},{\hat{y}}_{i}^{\left(t\right)}\right)+\overset{t}{\underset{i=1}{\sum }}\Omega \left(f_{i}\right), \end{array}$$

where *n* represents the number of trees, *l* is the training loss function, and *Ω* is the regularization term.

Then, the XGBoost takes the Taylor expansion of the loss function up to the second order and removes all the constants, so the specific objective at step *t* can be describes as

(56) $$\begin{array}{c} L^{\left(t\right)}=\Sigma_{\text{ⅈ}=1}^{n}\left[g_{i}f_{t}\left(x_{i}\right)+\frac{1}{2}h_{i}f_{t}^{2}\left(x_{i}\right)\right]+\Omega \left(f_{t}\right), \end{array}$$

where *g*_*i*_ and *h*_*i*_ can be described as follows:

(57) $$\begin{array}{c} \left\{\begin{array}{c} g_{i}=\partial_{{\hat{y}}_{\text{i}}^{\left(t-1\right)}}l\left(y_{i},{\hat{y}}_{i}^{\left(t-1\right)}\right),\\ h_{i}=\partial_{{\hat{y}}_{i}^{\left(t-1\right)}}^{2}l\left(y_{i},{\hat{y}}_{i}^{\left(t-1\right)}\right). \end{array}\right. \end{array}$$

The value of the objective function only depends on *g*_*i*_ and *h*_*i*_.

It can optimize every loss function, including logistic regression and pairwise ranking, and it is simple to parallel and can greatly enhance the program efficiency with a fast model exploration [76].

### 3.4. Evaluation Measure

After realizing HPV prediction, we need to use statistical test method to evaluate the efficiency of prediction model. Leave-one-out cross-validation (LOO-CV) is a more common method of Bayesian model and a special case of *k*-fold cross validation [77], because when *k* is equal to sample size *n*, and it can be regarded as *n*-fold cross validation.

HPV typing is a two or three classification problem. If the HPV model predicts a positive result (*P*) and the true result is also positive, it is called true positive (TP). If the predicted result is negative (*N*), the real result is also positive, which is called false positive (FP). The results can be calculated by the following formula:

(58) $$\begin{array}{c} \text{accuarcy}\left(\text{ACC}\right)=\frac{\text{TP}+\text{TN}}{\text{TN}+\text{FP}+\text{FN}+\text{TP}}, \end{array}$$

(59) $$\begin{array}{c} \text{specificity}=\frac{\text{TN}}{\text{TN}+\text{FP}}, \end{array}$$

(60) $$\begin{array}{c} \text{sensitivity}=\frac{\text{TP}}{\text{TP}+\text{FN}}. \end{array}$$

## 4. Conclusion

High-risk HPV accounts for a higher proportion of cervical cancer in the world. Therefore, the identification of high-risk HPV is of great significance for the treatment of some major cancers such as cervical cancer [78]. At present, there are common epidemiological detection techniques for HPV typing [79], such as nucleic acid imprinted in situ hybridization or dot blot hybridization, and the detection infection rate is about 10-20% [80]. In addition, there are test methods, such as polymerase chain reaction (PCR). All HPV types can be detected by PCR, and the detection infection rate is more than 40%. In addition to experimental methods, some computational methods have been proposed to predict HPV typing.

We summarize the mathematical models and prediction methods of the risk types of human papillomavirus, especially around the key steps such as feature extraction, feature selection, and prediction algorithms. From the above research papers, it can be found that the prediction accuracy of low-risk types is often higher than that of high-risk types. E7 performed better than other HPV proteins in low-risk experiments. However, E6 performs best among all HPV proteins for high-risk prediction and all types of prediction experiments, which is just consistent with experimental studies. E5, E6, and E7 proteins of high-risk HPV play an important role in disease progression and cancer [81]. Therefore, E6 protein sequence is more suitable for HPV high-risk prediction, and E7 protein sequence is more suitable for HPV low-risk prediction. However, there are some exceptions. In the reduced amino acid modes, L1 protein performs better in predicting high-risk HPV, while L2 protein is more suitable for low-risk HPV. These conclusions can provide a theoretical basis for subsequent research and guide the establishment of HPV typing models.

Mutations usually lead to cell dysfunction, cell death, and even cancer in higher organisms. Therefore, mutations in HPV protein may make the virus more easily induced or carcinogenic and increase the chance of reinfecting the host or fleeing the host immune system. For example, the carcinogenicity of HPV is mainly controlled by E6 and E7 proteins, which often produce internal variation. The mutation frequency of E6 in cancer is 20% ~90%, and that of E7 is 60% ~90% [82]. A study in Japan showed that the mutation of aspartate to glutamate (d25e) at position 25 of HPV16 E6 protein was related to the DRB1 ∗ 1502 allele of HLA II. This mutation is considered to be an important mutation in invasive cancer and cervical intraepithelial neoplasia. In the Netherlands, the frequency of HLV DRB1 ∗ 07 allele increased in cancer patients with l83v mutation (*P* = 0.08). If the information of mutation information is considered in HPV classification model, it is also an effective way to improve HPV typing detection.

## Data Availability

HPV database can be downloaded from Los Alamos National Laboratory (LANL, https://lanl.gov).
